# Oroxylin a Inhibits the Protection of Bone Marrow Microenvironment on CML Cells Through CXCL12/CXCR4/P-gp Signaling Pathway

This article has been retracted.

**DOI:** 10.3389/fonc.2019.00188

**Published:** 2019-04-03

**Authors:** Hanbo Cao, Wenjun Li, Yizhou Zhou, Renxiang Tan, Yue Yang, You Zhou, Qinglong Guo, Li Zhao

**Affiliations:** ^1^State Key Laboratory of Natural Medicines, Jiangsu Key Laboratory of Carcinogenesis and Intervention, China Pharmaceutical University, Nanjing, China; ^2^State Key Laboratory Cultivation Base for TCM Quality and Efficacy, Nanjing University of Chinese Medicine, Nanjing, China

**Keywords:** bone marrow environment, CXCL12/CXCR4, oroxylin A, Imatinib (IM), β-catenin/P-gp

## Abstract

Imatinib (IM) resistance could have significant impact on the survival time of the CML-patients treated with IM. Previous studies have shown that the protective effects of the bone marrow stroma cells (BMSCs) on CML cells are achieved by the secretion of CXCL12. The aim of this study was to investigate whether Oroxylin A could reverse the protective effect of BMSCs on CML cells and illuminate the underlying mechanisms. The results showed that CXCL12 could enhance the resistance potential of K562 and KU812 cells to IM by increasing the expression of CXCR4, thus promoting the translocation of β-catenin into nucleus and subsequently increasing the expression of P-gp in K562 and KU812 cells. What's more, IM resistance could also be partially reversed by CXCR4 siRNA transfection. Moreover, the reverse effect of IM resistance by Oroxylin A was demonstrated by the inhibition of β-catenin/P-gp pathway via the decrease of CXCR4 *in vitro*. The *in vivo* study also showed that Oroxylin A could decrease the expression of P-gp and β-catenin in mice bone marrow with low toxicity, which could be consistent with the mechanisms verified *in vitro* studies. In conclusion, all these results showed that Oroxylin A improved the sensitivity of K562 and KU812 cells to IM in BM microenvironment by decreasing the expression of CXCR4 and then inhibiting β-catenin/P-gp pathway.

## Introduction

Chronic myeloid leukemia (CML), characterized by myeloproliferative disorder, represents 20% of all adult leukemia (1). Originating from the hematopoietic stem cell, CML is featured by the mutation of translocation of chromosomes 9q34 and 22q11 at cytogenetic level (2), leading to the formation of the fusion gene, BCR-ABL, which encodes a cytoplasmic protein with high tyrosine kinase activity (3).

BCR-ABL being validated as a target of CML, BCR-ABL specific tyrosine kinase inhibitors (TKIs), Imatinib (IM), Nilotinib, and Dasatinib, have been widely used in clinic. These substances can generate complete cytogenetic response (CCR) and largely abate BCR-ABL transcript levels (1, 4). Development of the drug IM is a crucial step in the treatment of patients with CML, especially in the chronic phase of the disease (5). However, resistance to IM occurs in the treatment process, developing in about 30% of patients via intrinsic or extrinsic factors. Intrinsic factors, such as acquisition of point mutations in BCR-ABL gene (e.g., T315I, F317L, F359C/V, G250E, Q252H, and E255K/V) accounts for ~50% of IM-resistance cases (6). Extrinsic factors, such as cytokines, growth factors, and matrix proteins, are mainly secreted by cells in the bone marrow (BM) microenvironment, serving to protect CMLs from TKIs attack (7).

The mechanisms of TKI resistance in CML cells are complicated, with some of them being even unclear. One of the most common causes of the resistance is the mutations in the BCR-ABL gene, which results in the failure of therapeutic response to TKIs. Another proposed mechanism, known as multidrug resistance, is generated by an insufficient drug concentration at the intracellular level. One of the reasons for this phenomenon may be due to the process of active transportation, a result of over-expression of the ABC-transporters P-glycoprotein (P-gp, encoded by the MDR1/ABCB1 gene), and/or breast cancer resistant protein (BCRP, encode by ABCG2 gene) (8, 9). MDR1 transports a large variety of endogenous substances and xenobiotics across extra- and intracellular membranes (10).

The BM microenvironment is demonstrated to have played a dominating role in the differentiation, migration, proliferation, survival, and drug resistance of leukemia cells, serving as a safe haven for normal and malignant hematopoietic cell. Specifically, in CML cells, BM microenvironment prevents them from TKIs-induced apoptosis (11, 12). BM stroma and stroma-derived factors are thought to play an important role in CML and other hematological malignancies, such as multiple myeloma and lymphoma (13–24). CXCL12, also recognized as stromal cell-derived factor-1 with subtypes of SDF-1α and SDF-1β, is a chemokine mainly produced by bone marrow stromal cells (BMSCs). It acts through the cognate chemokine receptor CXCR4 and CXCR7, to mediate homing, survival and proliferation of tumor cells, which contributes to soluble factor-mediated drug resistance. CXCR4, a seven-transmembrane G-protein-coupled chemokine receptor, is expressed by hematopoietic and epithelial cancer cells (25). The binding of CXCL12 to CXCR4 activates PI3K, one of downstream effectors of CXCR4, conferring drug resistance on cancer cells through PI3K/Akt/β-catenin pathway (26). Considering the close connection between BM and the drug resistance in CML cells, blocking of their interaction has been widely used as a therapeutic strategy. For example, the microenvironment protection for leukemic cells from chemotherapeutics-induced apoptosis could be abolished by CXCR4 antagonists such as plerixafor (AMD3100) (27).

Oroxylin A (C_16_H_12_O_5_, OA) is a bioactive flavonoid extracted from *Scutellaria baicalensis Georgi*, a herb used in the Traditional Chinese Medicine (28). Oroxylin A possesses a wide range of medical usage, including anti-inflammation, anticancer antiviral, and antibacterial infections (28). Our previous studies showed that Oroxylin A combined with Paclitaxel reverses cell adhesion mediated-drug resistance (CAM-DR) in HepG2 cells by inhibiting integrinβ1 and PI3K/Akt signaling (29). Furthermore, Oroxylin A could reverse multi-drug resistance in human hepatoma BEL7402/5-FU cells via down-regulation of P-glycoprotein expression by sabotaging NF-kB signaling pathway (30).

Also, our previous studies has demonstrated that Oroxylin A was able to reverse IM resistance in CML cells by inhibiting the CXCR7/ERK pathway, CXCR4/PI3K/Akt/NF-κB pathway and blocking the expression of P-gp by suppressing Stat3 pathway in the co-cultured group (31–33). In this research, we look forward to further exploring Oroxylin A's effect on CXCR4 in IM resistance of CML cells co-cultured with human bone marrow stromal cells (BMSCs). Then we investigated whether Oroxylin A could reverse the drug resistance by inhibiting CXCL12/CXCR4 axis, especially through suppressing PI3K/Akt/β-catenin/P-gp pathway.

## Results

### Human BM Environment Protects CML Cells From IM

A co-culture model was established by employing the human bone marrow stromal cells (hBMSCs) (34), aiming at simulating bone marrow microenvironment. Annexin V/PI assays and Ki67 expression were applied to evaluate the co-culture model. As was shown in Figures 1A,B,K562 and KU812 were less sensitive to IM in co-culture conditions for 48 h compared with those in normal conditions. Apoptosis rate in co-culture models was less than nor-culture after treatment of 4 μM IM (Figure 1A). Moreover, the Ki67 expression level in normal culture cells was lower than that in co-culture group. Meanwhile, the expressions of cleaved caspase-3 and caspase-9 after IM treatment were tested by western blotting assay. The activated form of caspase-3 and caspase-9 were obviously decreased in co-culture group compared with that in normal group, which further demonstrated that the BMSC cells protected CML cells from the damage caused by IM (Figures 1C,D). Therefore, these results showed that human BM environment not only protected CML cells from IM induced apoptosis but resulted in a stronger proliferative effect.

**Figure 1:** BM microenvironment protected CML cells from IM attack. K562 and KU812 cells were cultured with or without hBMSCs and with or without 4 μM IM for 48 h. Cell proliferation was determined by Annexin V-PI double-staining assay and Ki67 cell proliferation detection. **(A)** Apoptosis rate of K562 and KU812 after treatment by IM with or without hBMSCs. **(B)** Ki67 cell proliferation detection of K562 cells after treatment. **(C)** The expression of cleaved-caspase3 and 9 was determined using western blot analysis. **(D)** Analysis of proteins expression. Data **(A)** and **(D)** were shown as Means ± SD for three independent experiments (^*^p < 0.05 and ^**^p < 0.01).

### CXCL12 Secreted by BMSCs Activates CXCR4 Pathway in CML Cells

*In vivo*, the protective effect of BMSCs on CML cells is mainly due to the secretion of CXCL12 by BMSCs, which activate CXCR4 by its interaction with CXCR4, thus promoting the survival rate of CML cells (35). In co-culture system, the concentration of CXCL12 in upper medium was higher than that in normal-culture condition. We also find that the secretions of CXCL12 both in K562 and KU812 cells were in a time-dependent manner when co-cultured with hBMSCs (Figure 2A). With the presence of anti-CXCL12 (Neutralizing antibodies against SDF-1α) in the co-culture group, the expression of CXCR4 in K562 and KU812 cells was decreased in comparison to co-culture group without anti-CXCL12 (Figures 2B,C). Meanwhile, the expressions of the proteins regulated by CXCR4, such as PI3K, p-AKT, p-GSK3β, and β-catenin, were increased in the co-cultural group (Figures 2D,E). IF assay were further conducted to prove the nuclear-translocation of β-catenin in K562 cells (Figure 2F). The nuclear translocation of β-catenin was demonstrated to be more observable in co-culture group than that in normal culture group. The data suggested that co-culturing with human BMSCs could activate the nuclear-translocation of β-catenin. These results highlighted that CXCL12 secreted by BMSCs could activate CXCR4 pathway and induce nuclear translocation of β-catenin.

**Figure 2:** BM microenvironment stimulated CXCL12 secretion and activates CXCR4 in CML cells. K562 and KU812 cells were cultured with or without hBMSCs for 24 h or 48 h. **(A)** ELISA assay detection of CXCL12 secretion in CML cells co-cultured with BMSCs. **(B)** Western blot analysis of expression after cells co-cultured with BMSCs and Neutralizing CXCL12 (10 μg/ml). **(C)** Analysis of proteins expression. **(D)** The expression of downstream protein of CXCR4 was analyzed by western blot analysis. **(E)** Analysis of proteins expression. **(F)** Immunofluorescence detection of the distribution of β-catenin in K562 cells. Data **(A,C,E)** were shown as Means ± SD for three independent experiments (^*^p < 0.05 and ^**^p < 0.01).

### The Expression of P-gp Regulated by CXCR4/β-Catenin Pathway

To further identify the responsibility of CXCL12/CXCR4 pathway for the failure of IM treatment, a variety of proteins in ABC transporter family were detected by Western blot assay. Surprisingly, we found that P-gp expression was elevated in co-culture model while BCRP and MRP remained unchanged (Figures 3A,B). Silencing CXCR4 by siRNA not only impeded the expression of CXCR4, but the expression of β-catenin and P-gp as well. AMD3100, a pharmacological inhibition of CXCR4 by blockade of the interaction of CXCL12 and CXCR4, also suppressed the expression of β-catenin and P-gp (Figures 3C,D). Additionally, the degree of intracellular accumulation of Rh-123, was gauged by its fluorescence intensity measurement (Figure 3E). After being cultured with hBMSCs for 48 h, the Rh-123 accumulation in K562 and KU812 cells were reduced compared with normal culture, which suggested that BM mediated the convergence of P-gp activity. While in the AMD3100 and siRNA-CXCR4 group, the accumulation of Rh-123 were increased (Figure 3E), which suggested us CXCL12/CXCR4 axes contributed to IM resistance in human BM microenvironment.

**Figure 3:** The nuclear-translocation of β-catenin could regulate P-gp. **(A)** Western blot analysis in K562 cells co-cultured with hBMSCs for 48 h. **(B)** Western blot analysis of BCRP, MRP and P-gp. **(C,D)** Western blot analysis and **(E)** Intracellular Rh-123 fluorescence detection after K562 cells being treated with AMD3100 or CXCR4 Si RNA and co-cultured with or without BMSCs. **(F,G)** Western blot analysis of β-catenin in CML cells in nuclear and cytoplasm, respectively, and **(H)** immunofluorescence detection of the distribution of β-catenin in K562 and KU812 cells treated with LiCl. MDR1 mRNA and protein expression was detected by **(I)** RT-PCR assay and **(J,K)** western blot analysis in K562 and KU812 cells treated with LiCl or 20 μM Indo. Data **(B,E,G,I,K)** were shown as Means ± SD for three independent experiments (^*^p < 0.05, ^**^p < 0.01, and ^##^*p* < 0.01).

The results above showed that CXCR4 promoted the nuclear translocation of the β-catenin, and elevated the expression of P-gp. We purposed to explore the relationship between P-gp and β-catenin. LiCl, an activator of β-catenin, can enhance the expression and translocation of nuclear β-catenin. Conversely, indometacin (Indo), the inhibitor of β-catenin, has the opposite effect. As shown in Figures 3F–H, activating β-catenin either by employing LiCl or cultivating with BMSCs could enhance the mRNA and protein expression of P-gp. On the other hand, Indo had reversed effect (Figures 3I–K). Taken together, we believed that β-catenin could regulate, to some extent, the expression of P-gp.

### Oroxylin a Could Increase the Sensitive of CML Cells in Human BM Environment to IM

To evaluate the effect of Oroxylin A, cell apoptosis and proliferation assays were carried out in single/independent treatment or combined with IM. According to our previous research, 60 μM Oroxylin A harbored little cytotoxicity and its inhibition rate to K562 is < 5% (32). So 60 μM was chosen for the further tests. In co-cultural group treated with IM and Oroxylin A, apoptosis rate of K562 cells was increased. Similar circumstance was observed in KU812 cells (Figure 4A). The expression of Ki67 in combination group was less than that in IM alone (Figure 4B). Further results showed that the level of cleaved-caspase 3 and cleaved-caspase 9 were augmented in combination group compared with the IM alone group (Figures 4C,D). These results were also in accordance with our theory that Oroxylin A could reserve the resistance to IM in CML cells co-cultured with BMSCs.

**Figure 4:** Oroxylin A reversed the effect of protection of BMSCs on CML cells. K562 and KU812 cells were cultured with or without IM and Oroxylin A in normal group or co-culture group for 48 h. Cell proliferation was determined by Annexin V-PI double-staining assay and Ki67 cell proliferation detection. **(A)** Percentage of apoptosis in K562 and KU812 cells after treatment. **(B)** Ki67 cell proliferation detection. **(C)** The expression of cleaved-caspase3 and 9 was determined using western blot analysis. **(D)** Analysis of proteins expression. Data **(A)** and **(D)** were shown as Means Å SD for three independent experiments. (^*^p < 0.05 and ^**^p < 0.01).

### Oroxylin a Could Inhibit CXCR4/β-Catenin/P-gp Pathway in CML Cells Cultured in Human BM Environment

To further study the mechanism of the reversal effect of Oroxylin A, we performed Flow cytometer assay to detect the activation of CXCR4. Figure 5A showed that the increased function of CXCR4 caused by CXCL12/CXCR4 interaction was suppressed by Oroxylin A in K562 and KU812. Meanwhile, WB results showed that when CML cells were treated with Oroxylin A under co-culture conditions, the expression of CXCR4, β-catenin and P-gp was reduced significantly (Figures 5B,C). Then we explored the specific mechanism of Oroxylin A reversing the cyto-protective effect of bone marrow microenvironment on CML cells. Immunofluorescence experiments showed that Oroxylin A down-regulated the nuclear-translocation of β-catenin under co-cultural conditions (Figure 5D). As shown in Figure 5E, the Rh-123 accumulation was increased in co-culture group treated with IM and Oroxylin A, which suggested that Oroxylin A functioned to suppress P-gp activity. To sum up, Oroxylin A could increase the sensitivity of CML cells to IM in human BM microenvironment by inhibiting CXCR4/β-catenin/P-gp pathway.

**Figure 5:** The CXCR4/β-catenin/ P-gp contributed to the reversal effects of Oroxylin A on IM-resistant CML cells. CML cells treated with Oroxylin A in co-culture model. **(A)** Flow cytometry analysis of 12G5 in K562 and KU812 cells. **(B)** Western blot analysis of expression of CXCR4, β-catenin, and P-gp in K562 and KU812 cells. **(C)** Analysis of proteins expression. **(D)** Immunofluorescence detection of the distribution of β-catenin in K562 and KU812 cells. **(E)** Intracellular Rh-123 fluorescence measurement in co-culture model cells treated with IM alone or combination with Oroxylin A. Data were shown as Means ± SD for three independent experiments (^*^p < 0.05, ^**^p < 0.01, and ^##^*p* < 0.01).

### Oroxylin a Breaks the Protective Effect of Bone Marrow on CML Cells by Inhibiting the CXCR4/β-Catenin/P-gp Pathway *in vivo*

To investigate the sensibility of Oroxylin A with IM *in vivo*, we established a model of CML mice. In the experimental process, the weight of mice remained stable in combination group compared to IM alone (Figure 6A). Also, the treatment of IM combined with Oroxylin A dramatically increased the survival period of the experimental animals. As shown in Figure 6B, in the K562 transplantation group and co-transplantation group, mice death began from 23 days after being engrafted. The co-transplanted mice treated with IM alone began to die from/Day 40. While in the co-transplantation group, mice began to die from/Day 63 after Oroxylin A was combined with IM treatment. To further validate the anti-tumor effect of Oroxylin A, spleen was excised and weighed. In the spleens of the mice in negative control group splenomegalia was observed significantly at 9 weeks after transplantation. The weight increase of spleens was modified by combination treatment compared with IM treatment alone group (Figures 6C,D). To illuminate the potential mechanisms of Oroxylin A in combination with IM against leukemic cells *in vivo*, immunohistochemistry was performed. CD45, the marker of leukocytes, was detected to indicate the leukemia cells in bone marrows. As shown in Figure 6E, Co-treatment of IM and Oroxylin A synergistically reduced the expression of CD45 in mice bone marrow when compared with IM alone. The results showed us that Oroxylin A and IM are synergistic to inhibit cell proliferation of K562 cells. This mechanism was verified by IHC assay. We also found that the expression of CXCR4, β-catenin and P-gp was increased in co-transplanted group compared with control group in thigh bones, which caused the drug-resistance of IM. Although IM itself was able to lower these proteins in co-transplanted group, Oroxylin A significantly augmented its ability in reducing the expression. In summary, the CXCR4/β-catenin/ P-gp pathway was activated in our co-transplanted model *in vivo* and Oroxylin A could reverse the activation effect.

**Figure 6:** The reversal effect and mechanisms of Oroxylin A *in vivo*. Tumor xenografts inoculated with K562 cells or combinations with hBMSCs were treated with IM (200 mg/kg) or combination with Oroxylin A (80 mg/ kg) every other day orally for 4 weeks. **(A)** The analysis of body weight after indicated. **(B)** Survival Curves of mice after different treatment. **(C)** The weight of spleens of treatment groups. **(D)** Images of representative spleens. **(E)** Representative IHC staining of murine BM, for human CD45, β-catenin and P-gp antigen.

## Discussions

The present study demonstrated that BM environment induced CML cells resistance to IM through activation of CXCL12/CXCR4/β-catenin/P-gp pathway, while Oroxylin A potentiate the anti-leukemia activity of IM to CML cells by interfering with CXCL12/CXCR4 activation and inhibiting the expression of P-gp *in vitro* and *in vivo*.

Based on our previous researches, this study focused on the function of CXCL12/CXCR4 axis in the drug resistance phenomenon of CML cells to IM in BM environment. In this article, we established BM environment model and induced CML drug-resistance by co-culturing CML cells with human BMSCs. The results showed that the sensitivity of CML cells to IM was significantly reduced in co-culture models, which was ascribed to the secretion of CXCL12 and activation of the downstream signaling. CXCR4, the receptor of CXCL12, is connected with the metastasis and progression of leukemia in clinic trails. It has been reported that the activation of CXCR4 in leukemia cells promotes cell survival, metastasis and other processes through CXCR4's downstream pathways, like PI3K/AKT/FOXO3α, ERK/MAPK, NF-κB, and STAT3 (36, 37). In this study, CXCR4 facilitates the nuclear translocation of β-catenin by activating PI3K/AKT pathway and by increasing the expression of GSK3β. In addition, Oroxylin A can also reverse this effect through blocking the interaction between BM and CML.

Most patients with advanced cancer deceased for the develop resistance to available therapies (38–40). P-gp is one of the factors contributing to these mechanisms. In this research, we found that the expression of P-gp had a significantly higher level when stimulated by BM, which was a result of the activation of PI3K/AKT/β-catenin pathway, contributing to IM resistance. The expression of MDR1 mRNA and P-gp protein was increased when β-catenintranslocation into nuclear took place. However, additional Oroxylin A treatment was able to reverse the increased expression of P-gp in CML cells so as to enhance the sensitivity of cells to IM. Since the odds of other factors participating in the modulation of P-gp were not ruled out, we still need to explore the exact mechanism of P-gp's modulation in CML cells in the future.

Nowadays, in the treatment of various diseases, transplantation of MSCs is widely used, such as producing a local immunoprivileged site, engraftment of UCBT (umbilical cord blood transplantation), and prevent rejection and promote kidney transplantation tolerance (41–43). Basing on those reports, we established a model by co-transplantation of BMSCs and CML cells, allowing BMSCs to secrete CXCL12, thus aiming to discover the protective effect of human BM environment on CML. The mice model of CML used before varied according to different purposes, for example, we gained solid tumor models directly by subcutaneous injection, we inoculate the CML cells via tail vein and transfer the primary BM cells retro-virally transduced with p210Bcr-Abl into B6 mice intravenously according to the standard BM transplantation (BMT) procedure (32, 44). Based on these aspects, we established co-cultured animal models to verify the function of CXCL12. Our results demonstrated that the content of CXCL12 in mice with co-transplantation were higher than those without (data not shown). Meanwhile, we also verified that the interaction of BMSC cells and CML cells in mice contributed to a similar effect to that in the co-cultural model *in vitro*. Admittedly, this mice model needs to be improved and many other mechanisms, like the distribution of these cells in mice, need to be confirmed. Taking all these into consideration, this model is worth exploring in the future.

Oroxylin A shows effective anticancer activities and low-toxicities both *in vivo* and *in vitro*. Particularly, it can reverse drug resistance of many chemotherapeutical medicines, such as 5-FU, adriamycin, and paclitaxel (29, 33, 45), in several cancer cell lines, including CML cells. In this study, the potentiality of Oroxylin A in reversing protective effect of BMSCs was further confirmed. Moreover, Oroxylin A's effect on CML cells was partly attributed to the blocking of β-catenin translocation to nucleus and decreasing P-gp transcription, a possible target gene of β-catenin. The results *in vivo* also highlighted the possibility of treatment of Oroxylin A in combination with IM. These results indicated that Oroxylin A could be used as a CXCR4 inhibitor.

In this article, our study demonstrated that the activation of CXCL12/CXCR4 pathway was correlated with BM microenvironment and IM resistance in CML cells. Oroxylin A has been shown to potentiate the activity of IM against CML cells in the co-culture model. The mechanisms of Oroxylin A on improving the sensitivity of CML cells to IM might be related to the suppression of CXCL12/CXCR4 axis and its downstream pathway, Akt/GSK3β/β-catenin/ P-gp, *in vitro* and *in vivo*. In conclusion, Oroxylin A could be a novel and potent agent combined with IM for eradicating leukemia MDR.

## Materials and Methods

### Reagents and Antibodies

Oroxylin A (Oroxylin A purity>99%) was prepared at China Pharmaceutical University (Nanjing, China). The compound was dissolved in dimethyl sulfoxide (DMSO) (Sigma–Aldrich, St. Louis, USA) to a concentration of 100 mM and stored at −20°C. The culture medium was RPMI-1640 and DMEM/F12 (1:1) (Gibco, Invitrogen Corporation, Carlsbad, CA). Dye DAPI (Invitrogen, USA) was used to detected apoptosis cells. The final DMSO concentration did not exceed 0.1% throughout the study. Primary antibodies against GAPDH (1:10,000) and CXCR4 (1:1,000) were products from Bioworld (OH, USA). Primary antibodies against caspase3 (1:1,000), caspase9 (1:1,000), β-catenin (1:1,000), P-gp (1:1,000), PI3K (1:1,000), Akt (1:1,000), p-Akt (1:1,000), GSK3β (1:1,000) and p-GSK3β (1:1,000) were obtained from Cell Signaling Technology (Danvers, MA). Primary antibody against Actin (1:10,000) was obtained from Santa Cruz Biotechnology (Santa Cruz, CA). HRP Goat Anti-Rabbit lgG and Anti-Mouse lgG (1:20, 000,) was purchased from ABclonal (ABclonal, China). Imatinib was purchased from Melonepharma (Dalian, China). CXCR4 small interfering RNA (siRNA) was purchased from Santa Cruz Biotechnology, Inc (Santa Cruz, CA). LiCl was obtained from Sigma-Aldrich (Sigma-Aldrich, St. Louis, USA).

### BMSCs Isolation and Culture

Primary human BMSCs were isolated from the iliac crest BM aspirates of healthy donors after informed consent was obtained. The clinical sample collections complied with guidelines in the Declaration of Helsinki and were approved by Nanjing Drum Tower Hospital's institutional review board. All patients had signed the consent forms. BM mononuclear cells were isolated by Percoll (Solarbio), Dulbecco's modified Eagle's medium (DMEM) (Euroclone) with 1,000 mg/ml glucose and _L−_glutamine, centrifuged and plated at a density of 1,000 cells/cm^2^. BMSCs were cultured in L-DMEM/F12 (GIBCO, USA) with 15% fetal bovine serum (GIBCO) at 37°C with 5% CO_2_. Four days later, non-adherent cells were removed carefully and the culture medium was refreshed. When primary cultures became almost confluent, the culture was treated with 0.5 ml of 0.25% trypsin containing 0.02% mmol/L ethylenediamine tetraacetic acid (GIBCO, USA) for 4 min at room temperature (25°C). A purified population of BMSCs was obtained 1 week after the initiation of culture.

### Cell Line and Culture Conditions

Human CML cell line K562 and KU812 were purchased from Cell Bank of Shanghai Institute of Biochemistry & Cell Biology at September 2017. All cell lines were authenticated based on STR fingerprinting and last checked in August 2014. Cells were cultured in RPMI-1640 medium supplemented with 10% heat-inactivated fetal bovine serum (GIBCO, USA), in a humidified environment with 5% CO_2_ at 37°C.

### Annexin V/PI Staining

BMSCs were seeded in six-well plates (Corning, USA). After 12 h, K562 cells or KU812 cells were plated in the same plate. K562 cells or KU812 cells were harvested after Oroxylin A and IM treatment, and stained with the Annexin V/PI Cell Apoptosis Detection Kit (KeyGen Biotech, Nanjing, China) according to the manufacturer's instructions. Data acquisition and analysis were performed with a Becton Dickinson FACS Calibur flow cytometer using Flowjo 7 software at Ex./Em._488/530 nm.

### Western Blot Analysis

Cells were collected and lysed in lysis buffer (50 mM Tris–HCl, pH 7.6, 150 mM NaCl, 1 mM EDTA, 1% (m/v) NP-40, 0.2 mM phenylmethanesulfonyl fluoride (PMSF), 0.1 mM NaF, and 1.0 mM dithiothreitol). The lysates were centrifuged at 4°C for 30 min at 12,000 × g. The supernatant was used to determine the protein concentration by bicinchoninic acid (BCA) assay kit (Pierce, Rockford) with a Varioskan multimode microplate spectrophotometer (Thermo Waltham, MA, USA). Protein samples were loaded on 10% SDS–PAGE gel and transferred to nitrocellulose membranes (BioTrace NT, PallCor, USA). The membranes were then blocked with 1% BSA in PBS for 1 h, followed by incubating with primary antibodies at 4°C overnight. After three washes with PBST, the membrane was incubated with HRP Goat Anti-Rabbit lgG or Anti-Mouse lgG conjugated second antibody for 1 h at room temperature. Detection was performed with an Amersham Imager 600 RGB (GE, USA).

### DAPI Staining

BMSCs alone or co-cultured with CML cells were treated at indicated concentration of substances. After treatment, the cells were fixed with 4% paraformaldehyde (PFA) for 25 min, washed thrice with cold PBS for 5 min and incubated with 0.2% Triton X- 100 for 25 min, then stained with 1 mg/ml diamidino-phenyl-indole (DAPI) for 10 min, and washed thrice with cold PBS for 5 min. The nuclear morphology of cells was examined by fluorescence microscopy (OlympusIX51; Olympus Corporation, Tokyo, Japan) with a peak-excitation wave length of 340 nm.

### Rh-123 Accumulation

After treatment, CML cells were harvested and 5 μg/ml Rhodamine 123 (Rh-123, MedChemExpress, China) was incubated for 30 min. Cells were placed in ice water to cease the reaction followed by harvesting and twice-washing with ice-cold PBS. Then samples were analyzed by FACSCalibur (Becton–Dickinson). Excitation wave-length and emission wavelength are 488 and 530 nm, respectively.

### Immunofluorescence Confocal Microscopy

Treated CML cells were harvested and seeded onto glass coverslips specially prepared for immunofluorescence. After washing twice with cold PBS for 5 min, cells were fixed with 4% paraformaldehyde (PFA) for 25 min, and permeabilized with PBS containing 0.2% Triton X-100 for 25 min. Then, the cells were blocked with 3% BSA in PBS for 1 h, and incubated with anti-CXCR4 antibody (1:50) at 4°C overnight. After washing thrice with PBS for 5 min, the cells were stained with FITC-conjugated anti-rabbit IgG antibody (1:200) at 37°C for 1 h. After counterstaining with DAPI, (Invitrogen, USA) for 20 min, the images were captured with an Olympus FV1000 confocal microscope.

### Immunohistochemistry

Marrow samples were removed from both physiological saline and Oroxylin A and IM combination treated or alone. The expression of CD45^+^, CXCR4, P-gp, β-catenin were assessed by immunohistochemical method using a rabbit-anti-human monoclonal antibody and an Ultra-Sensitive™ SP kit (kit 9710 MAIXIN, Fuzhou, Fujian). Tissue sections (4 μm thick) were placed onto treated slides (Vectabond, Burlingame, California, US). Sections were heat fixed, deparaffinized and rehydrated through graded alcohols (100, 95, 85, and 75%). Tissue sections were boiled in citrate buffer at high temperature for antigen retrieval, and treated with 3% hydrogen peroxide to block endogenous peroxidase activity. The slides were incubated with a protein-blocking agent (kit 9710 MAIXIN, Fuzhou, Fujian) prior to the application of the primary antibody, and then incubated with the primary antibody at 4°C overnight. The tissues were then incubated with the secondary biotinylated anti-species antibody and labeled using a modification of the avidin–biotin complex immunoperoxidase staining according to the UltraSensitive™ SP kit manual. Counterstaining was done with Harris hematoxylin. Images were captured using a camera attached to computer.

### siRNA Transient Transfection

The transient transfection assay was carried out in 6-well plates using PepMute™ siRNA Transfection Reagent (SignaGen® Laboratories, USA) according to the manufacturer's instruction. First, PepMute™ transfection buffer was diluted before use, and then 3.3 μl siRNA in 1 ml RPMI 1640 medium was added gently and incubated for 15 min at room temperature. The complexes were added to each well and mixed gently by rocking the plates back and forth. The plates were then incubated at 37°C in a CO_2_ incubator. After 48 h, cells were collected for further experiments. The CXCR4 siRNA product was purchased from Santa Cruz Biotechnology, Inc. (Santa Cruz, CA).

### Animal Experiment

The animal study was carried out according to the regulations of China Food and Drug Administration (CFDA) on Animal Care. This study was reviewed and approved by Animal Care Use Committee of Jiangsu Province (Animal authorization reference number: SYXK2012-0035). Male NOD/SCID mice (35–40 days old, weighing 18–22 g) were supplied by the Model Animal Research Center of Nanjing University. The mice were raised in air-conditioned rooms under controlled lighting (12 h lighting/d) and were fed with standard laboratory food and water. We transplanted K562 cells combined with hBMSCs or K562 cells alone into NOD/SCID mice intravenously at 5 × 10^5^ and 2 × 10^5^ cells/mice, respectively. One week later, the increasing number of the leukocytes detected in the peripheral blood of vaccinated mice (data not shown), indicating that numerous CML cells had been engrafted into mice. The NOD/SCID mice with similar weight were randomly divided into six groups: negative control (normal mice), control (transplanted K562 cells), co-culture group (transplanted K562 and hBMS cells), IM monotherapy (transplanted K562 cells or co-transplanted), and combination group (treatment IM and Oroxylin A in co-transplanted) (*n* = 6). Four weeks later, the mice were treated with Oroxylin A (200 mg/kg), and IM (200 mg/kg) (Sigma Aldrich, US) alone or in combination. After treatment for 30 days, marrow contents of femurs and spleen were obtained. These sample cells were assessed by labeling with anti FITC-CD13 (eBioscience, California, US) antibody and analyzed by flow cytometry.

### Statistical Analysis

All data shown represent mean ± SD from triplicate experiments performed in a parallel manner unless otherwise indicated. All comparisons of data were made using Student's *t*-test and were considered to be statistically significant at *P* < 0.05.

## Data Availability

This manuscript contains previously unpublished data. The name of the repository and accession number are not available.

## Author Contributions

HC designed and performed experiments, analyzed date and wrote the paper. WL performed experiments and analyzed data. YiZ performed experiments. YY, RT, and YoZ provided relevant advice. QG and LZ oversaw the project, designed experiments, analyzed data and wrote the paper.

### Conflict of Interest Statement

The authors declare that the research was conducted in the absence of any commercial or financial relationships that could be construed as a potential conflict of interest.

## Abbreviations

CML: chronic myeloid leukemia
BM: bone marrow
h-BMSCs: human-bone marrow stromal cells
IM: Imatinib
TKIs: tyrosine kinase inhibitors
CCR: complete cytogenetic response
Indo: indomethacin.
